The article "Event-Triggered Finite-Time Attitude Cooperative Control for Multiple Unmanned Aerial Vehicles" was published in 2022. Journal: Appl Bionics Biomech.

# Event-Triggered Finite-Time Attitude Cooperative Control for Multiple Unmanned Aerial Vehicles

**DOI:** 10.1155/2022/5875004

**Published:** 2022-02-21

**Authors:** Qiang Han, Yongshuai Zhou, Xin Liu, Xianguo Tuo

**Affiliations:** ^1^Robot Technology Used for Special Environment Key Laboratory of Sichuan Province, Southwest University of Science and Techno1ogy 621010, China; ^2^Artificial Intelligence Key Laboratory of Sichuan Province, Sichuan University of Science & Engineering, Zigong 643000, China

## Abstract

The finite-time attitude cooperative control problem for a group of multiple unmanned aerial vehicle systems with external disturbances and uncertain parameters is discussed in this paper. The dynamics of the systems is described by quaternion avoiding the singularity. Based on the attitude error and angular velocity error, a novel nonsingular terminal sliding mode surface is proposed for the controller with event-triggered scheme. The lumped disturbances are estimated by neural networks with adaptive law. The communication frequency is decreased by the proposed distributed event-triggered based sliding mode controller. Lyapunov theory is utilized to analyze the stability of the systems, and the Zeno behavior is avoided by rigorous proof. Finally, simulation examples are presented to illustrate the efficiency of the proposed control algorithm.

## 1. Introduction

Attitude cooperative control of multiple unmanned aerial vehicle systems (MUAVs) is significantly important in the formation flying missions. Compared to a single unmanned aerial vehicle (UAV), MUAVs can accomplish more complex and dangerous missions by collaboration, such as search and rescue, forest fire fighting, emergency rescue, low-attitude reconnaissance, and combat military missions [1–3]. Attitude cooperative control problem has been of growing interests in last several years due to its engineering and theoretical implications. Many scholars proposed different attitude control scheme to improve the accuracy and stability of the MUAVs. Variable structure control combined with decentralized communication scheme was proposed for spacecraft formation flying [4], based on the development of consensus theory, leader-follower was employed in the multiple aircrafts [5, 6]. As the amount of the MUAVs increases, the communication burden among each UAV will increase and may cause the network communication jam, and it would seriously affect the stability of the systems due to the band width is limited. It is significant to consider the network communication strategy of MUAVs when designing the attitude cooperative controller.

Even-triggered scheme is employed in the multiagent systems for considering the limited band width and energy consumption, instead of continuous control input update, the controller updates the input depending on the event-triggered function, which is relevant to the measurement error, and when the estimation error comes up to the given threshold value the update of the controller will be updated [7]. An event-triggered-based controller was proposed in first-order multiagent systems (MAS) by introducing the event-triggered mechanism, and the triggered condition was designed associated with the states of agents [8]. Distributed rendezvous problem was investigated for second-order multiagent systems with combinational measurement by event-triggered mechanism [9]. Based on the measurement error, the event triggered function was built for linear MAS, and all the states of the agents reach to consensus [10, 11]. Event-triggered scheme was employed in many system dynamical model which can be described as second-order dynamics [12]. A distributed sliding mode controller based on event triggered finite time mechanism was designed for formation of multirobot systems [13]. The event triggered was widely used in attitude control of spacecrafts to save the communication resources [14–16]. However, the mentioned works with attitude control did not consider the uncertain parameters. Based on event-triggered strategy, time-varying formation problem was investigated for MUAVs under switching topology [17], attitude formation on SO (8) [18], and dynamical consensus formation problem which was limited by time-varying disturbances [19]. However, external disturbances and inertial matrix uncertainty cannot avoid in practical environment. The event-based formation control for MUAVs only guarantees asymptotically convergence in the aforementioned works [17–19]. Finite-time control is a useful tool which has high accuracy and robustness property, enabling the control systems to approach the stable region in finite time. Finite-time control has been extensively utilized in Euler-Lagrange systems [20–22]. Distributed attitude tracking problem of spacecrafts was proposed considering disturbances and uncertain parameters in finite time [20]. Adaptive control was introduced into the finite-time controller extended the mentioned work [20] for attitude tracking problem of spacecrafts [21]. Feedback control was employed in formation control for finite time convergence of nonholonomic wheeled mobile robots [22]. Distributed finite-time control (FTC) problem was studied for multiple quadrotor formation with the information of leader not available to all the followers [23]. However, no external disturbances were considered. The disturbance was estimated by the observer, and FTC was investigated for a single quadrotor [24, 25]. However, attitude cooperative problem was not considered. There is less work associated with the finite-time attitude cooperative or formation control with event-triggered mechanism for MUAVs. Most recently, FTC based on event-triggered was investigated for quadrotor flying control [26, 27]. However, attitude tracking problem was not considered, and the controller designed was limited to the specific UAV. So, attitude cooperative control with FTC theory and event-triggered mechanism is more interesting.

The article "Event-Triggered Finite-Time Attitude Cooperative Control for Multiple Unmanned Aerial Vehicles" was published in 2022. Journal: Appl Bionics Biomech.

Motivated by the aforementioned works and analysis, finite-time attitude cooperative control problem of MUAVs with event-triggered mechanism is investigated, and the network communication resources are reduced. The contribution of this paper is illustrated in the following aspects: (1) external disturbances and uncertain parameters are considered in the attitude dynamics, and the attitude cooperative problem is described by the quaternion avoiding the singularity. The attitude tracking consensus errors are measured by employing a positive error function, a novel integral sliding mode surface is proposed, the FTC is designed for the closed loop systems, and neural network is utilized to estimate the lumped uncertainties. (2) The communication frequency of the controller among the followers is reduced due to the event-triggered strategy which is employed in the controller, so the proposed novel event-triggered function saves the communication burden and energy of each UAV. The deduced lower bound between triggering intervals guarantee no Zeno behavior occurs. (3) Fast terminal sliding mode control is utilized in control law which guarantees that the attitude achieves the desired value in finite time.

The rest of this paper is organized as follows. In Section 2, preliminaries of graph theory, quaternion-based attitude dynamics of MUAVs, and some useful lemmas are given, and Section 3 gives main results. The performance of the controller is proved by numerical simulation examples in Section 4. Finally, conclusion is given in Section 5.

## 2. Preliminaries and Problem Formulation

### 2.1. Notations

The following convenience notations are adopted throughout the paper: *R*^*n*^ denotes *n* × 1 real column vector, *I*_*n*_ = [1, ...1]^*T*^ denotes *n* × 1 column vector with each element being, and *I*_*n*_ denotes a *n* × *n* dimensional identity matrix. ⊗ stands for Kronecker product. ‖.‖ stands for the induced matrix 2-norm or the Euclidean vector norm. In addition, for a given vector *x* ∈ *R*_*n*_, *x*_*i*_ denotes the *i*th element of the vector *x*, *sig*^*r*^(*x*) = sgn(*x*)|*x*|^*r*^.

The article "Event-Triggered Finite-Time Attitude Cooperative Control for Multiple Unmanned Aerial Vehicles" was published in 2022. Journal: Appl Bionics Biomech.

Graph theory is utilized to describe the communication flow among the MUAVs. Let *G* = (*ν*, *ξ*) denotes the graph, in which, *ν* = {*ν*_1_, *ν*_2_, ⋯, *ν*_*n*_} is a nonempty set containing a group number of nodes which denotes the UAV, and *ξ*⊆*ν* × *ν* is called edge which is a set of nodes. If there any two nodes could communicate with each other, the graph *G* is called connected graph. *A* = [*a*_*ij*_]_*N*×*N*_ ∈ *R*^*n*×*n*^ is weighted adjacency matrix representing the communication between each node, in which, *a*_*ii*_ = 0, otherwise, *a*_*ij*_ = *a*_*ji*_ ≥ 0. *D* = diag{*d*_1_, *d*_2_, ⋯, *n*} denotes the degree matrix of associated with weighted graph, the elements of the degree matrix are *d*_*i*_ = ∑_*j*=1_^*n*^*a*_*ij*_. The Laplacian matrix of the weighted graph is denoted by *L* = *D* − *A*, and *L* is symmetric matrix.

Throughout this paper, leader-follower MUAVs are considered which contains one leader and *n* followers. The followers are marked as *i*(*i* = 1, ⋯, *n*), and the leader is marked as 0. Let $\bar{G}$ denotes the topology graph associated with MUAVs containing one leader and *n* followers. A diagonal matrix *B* = diag{*b*_1_, ⋯, *b*_*n*_} is utilized to denote the communication between the follower UAV and the leader UAV. If *b*_*i*_ > 0 means that the *i*th follower can obtain the communication flow of the leader, otherwise, *b*_*i*_ = 0.

**Assumption 1 .**

Consider the MUAVs consisting of *N* followers and one leader, the topology of the MUAVs is described by $\bar{G}$, and $\bar{G}$ is directed connected graph.

Based on Assumption 1 and graph theory, we define a matrix *C* = *L* + *B*.

**Lemma 1 (see [28]).**

If Assumption 1 holds, then, matrix *C* is invertible.

**Lemma 2 (see [29]).**

Consider a system modeled as $\dot{z}=f\left(z\right),f\left(0\right)=0,x\in {\mathbb{R}}^{n}$, a continuous function *V*(*z*) ∈ *ℂ*^1^ which is defined on a neighbourhood of the origin. If the function *V*(*z*) satisfies that it is positive definite and $\dot{V}\left(z\right)\leq -\nabla_{1}V^{\partial }\left(z\right)$, where *∂* ∈ (0, 1), ∇_1_ is positive parameters. The systems converge to the origin in finite-time, the converge time *T* which depends on the initial state of *z*(0):

(1) $$\begin{array}{c} T\left(z\left(0\right)\right)\leq \frac{V^{1-\partial }\left(z\left(0\right)\right)}{\nabla_{1}\left(1-\partial \right)}. \end{array}$$

**Lemma 3 (see [30]).**

If there is a real number *x*_*i*_ ∈ ℝ, *i* = 1, ⋯, *n*, *α* ∈ (0, 1], then

(2) $$\begin{array}{c} {\left(\overset{n}{\underset{i=1}{\sum }}\;|\;x_{i}\;|\;\right)}^{\alpha }\leq \overset{n}{\underset{i=1}{\sum }}{\left|x_{i}\right|}^{\alpha }\leq n^{1-\alpha }{\left(\overset{n}{\underset{i=1}{\sum }}\;|\;x_{i}\;|\;\right)}^{\alpha }. \end{array}$$

For *x* ∈ ℝ^*n*^, |*α*| ∈ (0, 1), then

(3) $$\begin{array}{c} \left\|x^{\alpha }\right\|\leq n^{1-\alpha }{\left\|x\right\|}^{\alpha }. \end{array}$$

The article "Event-Triggered Finite-Time Attitude Cooperative Control for Multiple Unmanned Aerial Vehicles" was published in 2022. Journal: Appl Bionics Biomech.

### 2.2. Attitude Dynamics Model of MUAVs

Throughout this paper, the attitude dynamics of UAV is described by quaternion which could avoid singular problem and analyze conveniently [31].

(4) $$\begin{array}{c} J_{i}{\dot{\omega }}_{i}=u_{i}-S\left(\omega_{i}\right)J_{i}\omega_{i}+\vartheta_{i},\\ {\dot{Q}}_{i}=\frac{1}{2}\phi \left(Q_{i}\right)\omega_{i}, \end{array}$$

where *Q*_*i*_ = [*q*_*i*_ *q*_*i*0_]^*T*^ represents the attitude of the *i*th UAV, *q*_*i*_ ∈ ℝ^3^, *q*_*i*0_ ∈ ℝ, *Q*_*i*_ ∈ ℝ^4^, *Q*_*i*_ ∈ ℝ^4^, |*Q*_*i*_| = 1, and *ω*_*i*_ ∈ ℝ^3^ is the angular velocity. *J*_*i*_ denotes the inertia matrix of the *i*th UAV and is positive definite; *u*_*i*_ denotes the control torque of the *i*th UAV; *ϑ*_*i*_ denotes the external disturbances. *ϕ*(*Q*_*i*_) is given by

(5) $$\begin{array}{c} \phi \left(Q_{i}\right)=\left(\begin{array}{c} q_{i0}I_{3}+S\left(q_{i}\right)\\ -{q_{i}}^{Τ} \end{array}\right). \end{array}$$

For a vector given as *n* = [*n*_1_, *n*_2_, *n*_3_]^*T*^ ∈ *R*^3×1^, *S*(*n*) is defined as

(6) $$\begin{array}{c} S\left(n\right)=\left(\begin{array}{ccc} 0 & ‐n_{3} & n_{2}\\ n_{3} & 0 & ‐n_{1}\\ ‐n_{2} & n_{1} & 0 \end{array}\right). \end{array}$$

Let *R*(*Q*_*i*_) denote the rotation matrix which is given as *R*(*Q*_*i*_) = (2*q*_*i*0_^2^ − 1)*I*_3_ + 2*q*_*i*_*q*_*i*_^*T*^ − 2*q*_*i*0_*Π*(*q*_*i*_), *Q*_*i*_ = [*q*_*i*_ *q*_*i*0_]^*T*^ for the attitude control of UAV, the rotation matrix denotes the inertial frame of the *i*th UAV into the body frame. The multiplication between two unit quarternions is given by

(7) $$\begin{array}{c} Q_{1}⊙Q_{2}=\left(\frac{q_{10}q_{2}+q_{20}q_{1}+S\left(q_{1}\right)q_{2}}{q_{10}q_{20}-q_{1}^{T}q_{2}}\right), \end{array}$$

where *Q*_1_ = [*q*_1_ *q*_10_]^*T*^ and *Q*_2_ = [*q*_2_ *q*_20_]^*T*^.

In the leader-following MUAVs, the followers adjust itself attitude to be consistent with the attitude of the leader. The attitude tracking errors and angular velocity errors of the *i*th UAV are given as follows

(8) $$\begin{array}{c} {\tilde{Q}}_{i}=Q_{i}^{-1}⊙Q_{d}, \end{array}$$

(9) $$\begin{array}{c} {\tilde{\omega }}_{i}=\omega_{i}-R\left({\tilde{Q}}_{i}\right)\omega_{d}, \end{array}$$

where *Q*_*d*_≜[*q*_*d*_, *η*_*d*_]^*T*^ denotes the desired attitude which is given *Q*_*d*_≜[*q*_*d*_, *η*_*d*_]^*T*^, and the desired angular velocity is denoted by *ω*_*d*_. Based on the definition of the tracking errors, ${\tilde{\omega }}_{i}$ and ${\tilde{Q}}_{i}$ represent the attitude velocity tracking error and angular tracking errors, respectively.

The article "Event-Triggered Finite-Time Attitude Cooperative Control for Multiple Unmanned Aerial Vehicles" was published in 2022. Journal: Appl Bionics Biomech.

The attitude tracking error systems can be obtained,

(10) $$\begin{array}{c} J_{\text{i}}{\dot{\tilde{\omega }}}_{\text{i}}=-{\omega_{\text{i}}}^{\times }\cdot J_{\text{i}}\omega_{\text{i}}+u_{\text{i}}+T_{\text{i}}\cdot \left[\Pi \left({\tilde{\omega }}_{\text{i}}\right)\cdot R\left(Q_{\text{id}}\right)\cdot \omega_{d}-R\left(Q_{\text{id}}\right)\cdot {\dot{\omega }}_{d}\right], \end{array}$$

(11) $$\begin{array}{c} {\dot{\tilde{Q}}}_{i}=\frac{1}{2}\phi \left({\tilde{Q}}_{\text{i}}\right)\cdot {\tilde{\omega }}_{\text{i}}. \end{array}$$

**Assumption 2 .**

Three positive constants *d*_*m*_, *σ*_1_, *σ*_2_ exist and are satisfying |*d*_*i*_| ≤ *d*_*m*_, |*ω*_*i*_| ≤ *σ*_1_, and $\left|{\dot{\omega }}_{i}\right|\leq \sigma_{2}$, respectively.

**Assumption 3 .**

The inertia matrix ${\bar{J}}_{i}$ is known and nonsingular. Δ*J* denotes the uncertainties and is bounded.

**Lemma 4 (see [32]).**

Considering the system formulated as eqs. (10) and (11), for sliding mode surface $\kappa_{i}={\tilde{\omega }}_{i}+r_{1}q_{i}+r_{2}q_{i}^{c}$, where 0 < *c* < 1, *r*_1_ > 0, *r*_2_ > 0, for *i* = 1, ⋯, *n*. If the sliding mode surface reaches zero, then, ${\tilde{\omega }}_{i}=0,q_{0,i}=1$ and *q*_*i*_ = 0 can be reached in finite time, respectively.

## 3. Main Results

### 3.1. Event-Triggered Finite-Time Control Design

In this section, the control objective is to design a finite-time control law such that the angular velocity errors ${\tilde{\omega }}_{i}$ and the error quaternions ${\tilde{Q}}_{i}$ of the closed-loop system (10) and (11) can converge to small regions in finite time, respectively.

First, the sliding mode surface ${\bar{s}}_{i}$ is defined as

(12) $$\begin{array}{c} {\bar{s}}_{i}={\bar{J}}_{i}\left[{\tilde{\omega }}_{i}+k_{1}{\tilde{q}}_{i}+k_{2}{Τ}_{i}\left({\tilde{q}}_{i}\right)\right], \end{array}$$

with ${Τ}_{i}\left({\tilde{q}}_{i}\right)\left({\tilde{q}}_{i}\right)={\left[{Τ}_{i1}\left({\tilde{q}}_{i1}\right),{Τ}_{i2}\left({\tilde{q}}_{i2}\right),{Τ}_{i3}\left({\tilde{q}}_{i3}\right)\right]}^{T}\in R^{3\times 1}$,

(13) $$\begin{array}{c} {Τ}_{ij}\left({\tilde{q}}_{ij}\right)=\left\{\begin{array}{c} {\text{sig}}^{\ell }\left({\tilde{q}}_{ij}\right),\text{if }s_{ij}^{*}=0\text{ or }s_{ij}^{*}\neq 0,\left|{\tilde{q}}_{ij}\right|>ϒ,\\ \varpi_{1}{\tilde{q}}_{ij}+\varpi_{2}\text{si}{\text{g}}^{2}\left({\tilde{q}}_{ij}\right),\text{if }s_{ij}^{*}\neq 0,\left|{\tilde{q}}_{ij}\right|\leq ϒ \end{array}\right. \end{array}$$

where *i* = 1, ⋯, *n*, *j* = 1, 2, 3, *s*_*i*_^∗^ = [*s*_*i*1_^∗^, *s*_*i*2_^∗^, *s*_*i*3_^∗^]^*T*^, and $s_{i}^{*}={\tilde{w}}_{i}+k_{1}{\tilde{q}}_{i}+k_{2}{\text{sig}}^{r}\left({\tilde{q}}_{i}\right)$, where *k*_1_ and *k*_2_ are positive constants. Define ${\text{sig}}^{\iota }\left({\tilde{q}}_{i}\right)={\left[{\text{sig}}^{\iota }\left({\tilde{q}}_{i1}\right),{\text{sig}}^{\iota }\left({\tilde{q}}_{i2}\right),{\text{sig}}^{\iota }\left({\tilde{q}}_{i3}\right)\right]}^{T}$, *ι* ∈ (0, 1), *ϖ*_1_ = (2 − *r*)*ϒ*^*r*−1^, *ϖ*_2_ = (*r* − 1)*ϒ*^*r*−2^, *ϒ* is a small positive constant.

The article "Event-Triggered Finite-Time Attitude Cooperative Control for Multiple Unmanned Aerial Vehicles" was published in 2022. Journal: Appl Bionics Biomech.

To develop the control law, the following equations are derived from (10) and (11):

(14) $$\begin{array}{c} {\bar{J}}_{i}\left({\dot{\tilde{w}}}_{i}+k_{1}{\dot{\tilde{q}}}_{i}+k_{2}{\dot{Τ}}_{i}\left({\tilde{q}}_{i}\right)\right)=z_{i}+\delta_{i}+u_{i}, \end{array}$$

where

(15) $$\begin{array}{c} z_{i}=-S\left(w_{i}\right){\bar{J}}_{i}w_{i}+{\bar{J}}_{i}\left(S\left({\tilde{w}}_{i}\right)R\left({\tilde{Q}}_{i}\right)w_{d}-R\left({\tilde{Q}}_{i}\right){\dot{w}}_{d}\right)+k_{1}{\bar{J}}_{i}{\dot{\tilde{q}}}_{i}+k_{2}{\bar{J}}_{i}{\dot{\alpha }}_{i}\left({\tilde{q}}_{i}\right), \end{array}$$

(16) $$\begin{array}{c} {\dot{\alpha }}_{i}\left({\tilde{q}}_{i}\right)=\left\{\begin{array}{c} r\mathrm{diag}\left({\left|{\tilde{q}}_{ij}\right|}^{r-1}\right){\tilde{q}}_{i},\;\text{if}\;s_{ij}^{*}=0\;\text{or}\;s_{ij}^{*}\neq 0,\;\left|{\tilde{q}}_{ij}\right|>\phi ,\\ l_{1}{\dot{\tilde{q}}}_{i}+2l_{2}{\tilde{q}}_{i}\mathrm{sgn}\left({\tilde{q}}_{i}\right){\dot{\tilde{q}}}_{i},\;\text{if}\;s_{ij}^{*}\neq 0,\;\left|{\tilde{q}}_{ij}\right|\leq \phi , \end{array}\right. \end{array}$$

(17) $$\begin{array}{c} \delta_{i}=\vartheta_{i}-{\tilde{J}}_{i}{\dot{\tilde{w}}}_{i}-S\left(w_{i}\right){\tilde{J}}_{i}w_{i}+{\tilde{J}}_{i}\left[S\left({\tilde{\omega }}_{\text{i}}\right)R\left({\tilde{Q}}_{i}\right)\omega_{d}-R\left({\tilde{Q}}_{i}\right){\dot{\omega }}_{d}\right]. \end{array}$$

*δ*_*i*_ is the lumped disturbances containing model uncertainty and external disturbances.

By (12) and (14), we can obtain

(18) $$\begin{array}{c} {\dot{\bar{s}}}_{i}=z_{i}+\delta_{i}+u_{i}. \end{array}$$

Based on the sliding mode surface ${\bar{s}}_{i}={\bar{J}}_{i}\left[{\tilde{\omega }}_{i}+k_{1}{\tilde{q}}_{i}+k_{2}{Τ}_{i}\left({\tilde{q}}_{i}\right)\right]$, a novel integral sliding mode surface is proposed which is given as follows

(19) $$\begin{array}{c} s_{i}={\bar{s}}_{i}-\int_{0}^{t}x_{i}^{\eta }dt, \end{array}$$

where $x_{i}=-\sum_{j\in N_{i}}a_{ij}\left({\bar{s}}_{i}-{\bar{s}}_{j}\right)+b_{i}{\bar{s}}_{i}$, and *η* ∈ (0.5, 1) is strictly the ratio of positive odd numbers. The derivative of (19) is

(20) $$\begin{array}{c} {\dot{s}}_{i}={\dot{\bar{s}}}_{i}-x_{i}^{\eta }. \end{array}$$

An event-triggered finite-time sliding mode consensus controller is designed as follows

(21) $$\begin{array}{c} u_{i}\left(t\right)=x_{i}^{\eta }\left(t_{k}^{i}\right)-k_{3}\mathrm{sign}\left(s_{i}\left(t_{k}^{i}\right)\right)-k_{4}s_{i}\left(t_{k}^{i}\right)-z_{i}\left(t_{k}^{i}\right)-{\hat{\delta }}_{i}\left(t_{k}^{i}\right), \end{array}$$

where *k*_3_ and *k*_4_ are positive constants, respectively. For *t* ∈ [*t*_*k*_^*i*^, *t*_*k*+1_^*i*^), *t*_*k*_^*i*^ is the latest event-triggered time for the *i*th UAV, and the UAV only updates the control protocol at its own event-triggered time.

The article "Event-Triggered Finite-Time Attitude Cooperative Control for Multiple Unmanned Aerial Vehicles" was published in 2022. Journal: Appl Bionics Biomech.

An adaptive radial basis function neural networks (RBFNNs) scheme is proposed for the unknown disturbance *δ*_*i*_, as RBFNNs can estimate the unknown continuous functions *δ*_*i*_ and ensure tracking error ultimately converges to an adequately small compact. Illustrated in Figure 1, the adaptive RBFNNs can be written as

(22) $$\begin{array}{c} {\hat{\delta }}_{i}={\hat{W}}_{i}^{T}H_{i}\left(X_{\text{in}}\right), \end{array}$$

where ${\hat{\delta }}_{i}\in {\mathbb{R}}^{3}$ is the RBFNNs output vector, $X_{\text{in}}={\left[{{\tilde{q}}_{i}}^{T},{{\tilde{w}}_{i}}^{T}\right]}^{T}\in {\mathbb{R}}^{6}$ is the input vector of the RBFNNs, ${\hat{W}}_{i}\in {\mathbb{R}}^{J\times 3}$ is the weight vector, *J* > 1 is the nodes number of middle hidden layer, *H*_*i*_ = [*h*_*i*1_, ⋯,*h*_*iJ*_]^*T*^ ∈ ℝ^*J*^ is the basis function vector, and *h*_*iJ*_ is being the commonly used Gaussian functions, which is simplified as

(23) $$\begin{array}{c} h_{iJ}\left(X_{\text{in}}\right)=\exp\left(-\frac{{\left\|X_{\text{in}}-c_{iJ}\right\|}^{2}}{\sigma_{iJ}}\right), \end{array}$$

where *c*_*iJ*_ is the center of the receptive field, and *σ*_*iJ*_ is the width of the Gaussian function. There exists an optimal vector *W*_*i*_^∗^ such that

(24) $$\begin{array}{c} \delta_{i}=W_{i}^{*T}H_{i}\left(X_{\text{in}}\right)+\varepsilon_{i}, \end{array}$$

where *ε*_*m*_^*i*^ denotes the maximum value of the RBFNNs estimation error ‖*ε*_*i*_‖.

Let ${\tilde{W}}_{i}=W_{i}^{*}-{\hat{W}}_{i}$ denotes the vector of weight errors, and the adaptive weight update law are designed as

(25) $$\begin{array}{c} {\dot{\hat{W}}}_{i}={AH}_{i}\left(X_{\text{in}}\right)s_{i}^{T}, \end{array}$$

where *A* is a positive-definite symmetric matrix of gains.

The measurement error of the event-triggered mechanism is defined as

(26) $$\begin{array}{c} e_{i}\left(t\right)=x_{i}^{\eta }\left(t_{k}^{i}\right)-x_{i}^{\eta }\left(t\right)-k_{3}\mathrm{sign}\left(s_{i}\left(t_{k}^{i}\right)\right)+k_{3}\mathrm{sign}\left(s_{i}\left(t\right)\right)-k_{4}s_{i}\left(t_{k}^{i}\right)+k_{4}s_{i}\left(t\right)-z_{i}\left(t_{k}^{i}\right)+z_{i}\left(t\right)-{\hat{\delta }}_{i}\left(t_{k}^{i}\right)+{\hat{\delta }}_{i}\left(t\right). \end{array}$$

The article "Event-Triggered Finite-Time Attitude Cooperative Control for Multiple Unmanned Aerial Vehicles" was published in 2022. Journal: Appl Bionics Biomech.

### 3.2. Stability Analysis

In the following, the stability of the attitude cooperative under event-triggered adaptive RBFNNs control law is analyzed in detail.

**Theorem 1 .**

On the basis of Assumptions 1, and considering that the system (10) and (11) under the action of the controller (21) and the adaptive weight update law (25), the following event-triggered function is given as follows

(27) $$\begin{array}{c} Y\left(t\right)=\left\|e_{i}\right\|-k_{3}-k_{4}\left\|s_{i}\right\|+\rho_{i}, \end{array}$$

where *ε*_*m*_^*i*^ < *ρ*_*i*_ < *k*_3_, and when the event-triggered function *Y*(*t*) > 0, that is, ‖*e*_*i*_‖ > *k*_3_ + *k*_4_‖*s*_*i*_‖ − *ρ*_*i*_, the event is triggered. The *i*th UAV performs information interaction and update the control protocol at its own event-triggered time. And the system can achieve finite-time consensus under this action.

**Proof**

First, selecting the Lyapunov function as follows

(28) $$\begin{array}{c} V_{1}=\frac{1}{2}s_{i}^{T}s_{i}+\frac{1}{2}\text{tr}\left({\tilde{W}}_{i}^{T}A^{-1}{\tilde{W}}_{i}\right). \end{array}$$

Taking the derivative of (28), substituting (21) and (26) into the derivative, we can obtain

(29) $$\begin{array}{c} {\dot{V}}_{1}=s_{i}^{T}\left(e_{i}-k_{3}\mathrm{sign}\left(s_{i}\right)-k_{4}s_{i}+\delta_{i}-{\hat{\delta }}_{i}\right)+\text{tr}\left(-{\tilde{W}}_{i}^{T}A^{-1}{\dot{\hat{W}}}_{i}\right)\leq \left\|s_{i}\right\|\left\|e_{i}\right\|-k_{3}\left\|s_{i}\right\|-k_{4}{\left\|s_{i}\right\|}^{2}+s_{i}^{T}\left({\tilde{W}}_{i}^{T}H_{i}+\varepsilon_{i}\right)+\text{tr}\left(-{\tilde{W}}_{i}^{T}A^{-1}{\dot{\hat{W}}}_{i}\right)\leq \left\|s_{i}\right\|\left(\left\|e_{i}\right\|-k_{3}-k_{4}\left\|s_{i}\right\|+\varepsilon_{m}^{i}\right)+\text{tr}\left({\tilde{W}}_{i}^{T}H_{i}s_{i}^{T}\right)+\text{tr}\left(-{\tilde{W}}_{i}^{T}A^{-1}{\dot{\hat{W}}}_{i}\right). \end{array}$$

By the adaptive weight update law (25), it is obtained that

(30) $$\begin{array}{c} {\dot{V}}_{1}\leq \left\|s_{i}\right\|\left(\left\|e_{i}\right\|-k_{3}-k_{4}\left\|s_{i}\right\|+\varepsilon_{m}^{i}\right). \end{array}$$

When the event-triggered function *Y*(*t*) ≤ 0, ‖*e*_*i*_‖ ≤ *k*_3_ + *k*_4_‖*s*_*i*_‖ − *ρ*_*i*_,

(31) $$\begin{array}{c} {\dot{V}}_{1}\leq -\left\|s_{i}\right\|\left(\rho_{i}-\varepsilon_{m}^{i}\right)<0. \end{array}$$

According to the Lyapunov stability theory, it can be seen that under the action of the controller (21), the adaptive weight update law (25), and the event-triggered function (27), the sliding mode surface *s*_*i*_ can realize *s*_*i*_ = 0 and ${\dot{s}}_{i}=0$. By lemma 2, the reaching time is given as follows

(32) $$\begin{array}{c} t_{r}=\frac{\sqrt{2}V_{1}^{1/2}\left(0\right)}{\rho_{i}-\varepsilon_{m}^{i}}. \end{array}$$

Then, select the Lyapunov function as

(33) $$\begin{array}{c} V_{2}=\frac{1}{2}{\bar{S}}^{Τ}{\left[\left(L+B\right)⊗I_{3}\right]}^{Τ}\left[\left(L+B\right)⊗I_{3}\right]\bar{S}, \end{array}$$

where $\bar{S}={\left[{{\bar{s}}_{1}}^{T},\cdots ,{{\bar{s}}_{n}}^{T}\right]}^{T}$.

The article "Event-Triggered Finite-Time Attitude Cooperative Control for Multiple Unmanned Aerial Vehicles" was published in 2022. Journal: Appl Bionics Biomech.

Define

(34) $$\begin{array}{c} p_{i}=\underset{j\in n_{i}}{\sum }a_{ij}\left({\bar{s}}_{i}-{\bar{s}}_{j}\right)+b_{i}{\bar{s}}_{i},\\ P={\left[p_{1}^{Τ},\cdots ,p_{n}^{Τ}\right]}^{Τ}=\left(L+B\right)⊗I_{3}\cdot \bar{S}. \end{array}$$

Then, we can get

(35) $$\begin{array}{c} V_{2}=\frac{1}{2}P^{Τ}P. \end{array}$$

Let *S* = [*s*_1_^*T*^, ⋯,*s*_*n*_^*T*^]^*T*^, when ${\dot{s}}_{i}=0$, we know ${\dot{\bar{s}}}_{i}=x_{i}^{\eta }$, then$\dot{\bar{S}}=-{\left[\left(L+B\right)⊗I_{3}\cdot \bar{S}\right]}^{\eta }$.

Under Assumption 1 and Lemma 2, it can be obtained that *λ*_min_(*L* + *B*) > 0. And taking the derivative of (35), we can obtain

(36) $$\begin{array}{c} {\dot{V}}_{2}=-P^{Τ}\left[\left(L+B\right)⊗I_{3}\right]{\left[\left(L+B\right)⊗I_{3}\cdot \bar{S}\right]}^{\eta }=-P^{Τ}\left[\left(L+B\right)⊗I_{3}\right]P^{\eta }\leq -\lambda_{\min}\left(L+B\right)P^{Τ}P^{\eta }, \end{array}$$

Since the positive odd ratio parameter *η* ∈ (0.5, 1), and combined with Lemma 3, we can find

(37) $$\begin{array}{c} {\dot{V}}_{2}\leq -\lambda_{\min}\left(L+B\right)\left(\overset{3n}{\underset{i=1}{\sum }}{\left|p_{i}\right|}^{1+\eta }\right)\leq -\lambda_{\min}\left(L+B\right){\left({\left\|P\right\|}^{2}\right)}^{1+\eta /2}\leq -2^{1+\eta /2}\lambda_{\min}\left(L+B\right)V_{2}^{1+\eta /2}. \end{array}$$

According to Lemma 1, under the action of the controller (21), the state of the system can reach and remain on the sliding mode surface $\bar{S}=0$ within finite time. The settling time is *t*_*f*_.

(38) $$\begin{array}{c} t_{f}=\frac{V_{2}^{1-\eta /2}}{2^{1+\eta /2}\lambda_{\min}\left(L+B\right)\left(1-\eta /2\right)}. \end{array}$$

When $\bar{S}=0$, then ${\bar{s}}_{i}={\bar{J}}_{i}\left[{\tilde{w}}_{i}+k_{1}{\tilde{q}}_{i}+k_{2}\alpha_{i}\left({\tilde{q}}_{i}\right)\right]=0$, so ${\tilde{w}}_{i}+k_{1}{\tilde{q}}_{i}+k_{2}\alpha_{i}\left({\tilde{q}}_{i}\right)=0$. According to Lemma 4, we know ${\tilde{w}}_{i}⟶0$, ${\tilde{q}}_{i}⟶0$ in finite time will be satisfied.

Next, we need to analyze whether the system has a minimum event-triggered time interval strictly greater than zero, which means that there is no Zeno behavior. When the event-triggered function (27) satisfies *Y*(*t*) > 0, the event is triggered. Combining (26), we can see that between any two adjacent event-triggered moments, ‖*e*_*i*_‖ increases from zero to *k*_3_ + *k*_4_‖*s*_*i*_‖ − *ρ*_*i*_, therefore, when the growth rate is the fastest, the event-triggered time interval is the smallest. In this case, when the minimum time interval is a value greater than zero, it can be guaranteed that there is no Zeno behavior.☐

**Theorem 2 .**

The article "Event-Triggered Finite-Time Attitude Cooperative Control for Multiple Unmanned Aerial Vehicles" was published in 2022. Journal: Appl Bionics Biomech.

Based on Assumption 1, the system (10) and (11) under the action of the controller (21), the adaptive weight update law (25), and the event-triggered function (27), the system does not have Zeno behavior under any initial conditions.

**Proof**

Let $\beta_{i}\left(t\right)=k_{3}\mathrm{sign}\left(s_{i}\left(t\right)\right)+k_{4}s_{i}\left(t\right)+z_{i}\left(t\right)+{\hat{\delta }}_{i}\left(t\right)$, since the system (10) and (11) can achieve consensus under the action of the controller (21), the adaptive weight update law (25), and the event-triggered function (27), $\left\|{\dot{\beta }}_{i}\left(t\right)\right\|$ have upper bounds, which are taken as ${\left\|{\dot{\beta }}_{i}\left(t\right)\right\|}_{\max}$. And combining (26) to derive ‖*e*_*i*_‖ as follows

(39) $$\begin{array}{c} \;\frac{d\left\|e_{i}\right\|}{dt}\leq \left\|\frac{{de}_{i}}{dt}\right\|\leq \left\|\frac{d\left[-x_{i}^{\eta }\left(t\right)+\beta_{i}\left(t\right)\right]}{dt}\right\|\leq \left\|\frac{d}{dt}x_{i}^{\eta }\left(t\right)\right\|+\left\|{\dot{\beta }}_{i}\left(t\right)\right\|\leq \eta \left\|x_{i}^{\eta -1}\right\|\left\|{\dot{x}}_{i}\right\|+{\left\|{\dot{\beta }}_{i}\left(t\right)\right\|}_{\max}. \end{array}$$

Let *X* = [*x*_1_^*T*^, ⋯,*x*_*n*_^*T*^]^*T*^, we can obtain $\dot{X}=-\left(L+B\right)⊗I_{3}\cdot \dot{\bar{S}}$. When $\dot{S}=0$, $\dot{\bar{S}}=X^{\eta }$ will be satisfied, so $\dot{X}=-\left(L+B\right)⊗I_{3}\cdot X^{\eta }$. And according to Lemma 3, we know

(40) $$\begin{array}{c} \left\|x_{i}^{\eta -1}\right\|\leq \left\|X^{\eta -1}\right\|\leq {\left(3n\right)}^{2-\eta }{\left\|X\right\|}^{\eta -1},\\ \left\|{\dot{x}}_{i}\right\|\leq \left\|\dot{X}\right\|\leq \left\|\left(L+B\right)⊗I_{3}\cdot X^{\eta }\right\|\leq \left\|L+B\right\|\left\|X^{\eta }\right\|\leq {\left(3n\right)}^{1-\eta }\left\|L+B\right\|{\left\|X\right\|}^{\eta }. \end{array}$$

By (38) and (39), we can obtain

(41) $$\begin{array}{c} \;\frac{d\left\|e_{i}\right\|}{dt}\leq \eta {\left(3n\right)}^{3-2\eta }\left\|L+B\right\|{\left\|X\right\|}^{2\eta -1}+{\left\|{\dot{\beta }}_{i}\left(t\right)\right\|}_{\max}. \end{array}$$

Due to *X* = −*P* and $\left\|P\right\|=\sqrt{2}V_{2}^{1/2}\left(t\right)\leq \sqrt{2}V_{2}^{1/2}\left(0\right)$, we have

(42) $$\begin{array}{c} \;\frac{d\left\|e_{i}\right\|}{dt}\leq 2^{2\eta -1/2}\eta {\left(3n\right)}^{3-2\eta }\left\|L+B\right\|V_{2}^{2\eta -1/2}\left(0\right)+{\left\|{\dot{\beta }}_{i}\left(t\right)\right\|}_{\max}. \end{array}$$

For any *t* ∈ [*t*_*k*_^*i*^, *t*_*k*+1_^*i*^), *t*_*k*_^*i*^ is the latest event-triggered time for the *i*th UAV, the time interval *T*_*m*_^*i*^ = *t*_*k*+1_^*i*^ − *t*_*k*_^*i*^, and ‖*e*_*i*_(*t*_*k*_^*i*^)‖ = 0 at the event-triggered moment, and let $\lambda_{i}=2^{2\eta -1/2}\eta {\left(3n\right)}^{3-2\eta }\left\|L+B\right\|V_{2}^{2\eta -1/2}\left(0\right)+{\left\|{\dot{\beta }}_{i}\left(t\right)\right\|}_{\max}$, we can obtain

(43) $$\begin{array}{c} \left\|e_{i}\left(t\right)\right\|-\left\|e_{i}\left(t_{k}^{i}\right)\right\|=\left\|e_{i}\left(t\right)\right\|\leq \left(t-t_{k}^{i}\right)\lambda_{i}\leq T_{m}^{i}\lambda_{i}. \end{array}$$

When the event-triggered function (27) satisfies *Y*(*t*) > 0, the event is triggered, we have

(44) $$\begin{array}{c} \left\|e_{i}\left(t\right)\right\|>k_{3}+k_{4}\left\|s_{i}\right\|-\rho_{i}>k_{3}-\rho_{i}. \end{array}$$

Combining (41) and (42), we can know

(45) $$\begin{array}{c} T_{m}^{i}>\frac{k_{3}-\rho_{i}}{\lambda_{i}}. \end{array}$$

It can be concluded from (43) that the event-triggered time interval is strictly greater than zero, so there is no Zeno behavior.☐

The article "Event-Triggered Finite-Time Attitude Cooperative Control for Multiple Unmanned Aerial Vehicles" was published in 2022. Journal: Appl Bionics Biomech.

## 4. Example Simulation

Considering the system composed of four UAVs includes three follower UAVs and one leader UAV, and the leader node is marked as 0. The directed communication topology is shown in Figure 2. Hence, we have

(46) $$\begin{array}{c} L=\left[\begin{array}{ccc} 1 & -1 & 0\\ 0 & 1 & -1\\ -1 & 0 & 1 \end{array}\right]B=\left[\begin{array}{ccc} 1 & 0 & 0\\ 0 & 1 & 0\\ 0 & 0 & 1 \end{array}\right]. \end{array}$$

The actual inertia matrices are assumed to be

(47) $$\begin{array}{c} J_{1}=\left[\begin{array}{ccc} 15 & 1 & 1\\ 2 & 16 & 0.5\\ 0 & 0.5 & 14 \end{array}\right]J_{2}=\left[\begin{array}{ccc} 13 & 0.5 & 0\\ 1 & 15 & 0.5\\ 0 & 1.5 & 14 \end{array}\right]J_{3}=\left[\begin{array}{ccc} 14 & 1 & 2\\ 0 & 13 & 0\\ 2 & 1 & 15 \end{array}\right]. \end{array}$$

With the existence of model uncertainties and external disturbances, the nominal inertia matrices of the UAV are given by ${\bar{J}}_{1}={\bar{J}}_{2}={\bar{J}}_{3}=\mathrm{diag}\left({\left[20\;20\;20\right]}^{T}\right)$. Take the disturbances as

(48) $$\begin{array}{c} d_{1}={\left[0.1\sin\left(t\right),0.2\cos\left(0.5t\right),0.15\cos\left(0.7t\right)\right]}^{T},\\ d_{2}={\left[0.1\cos\left(t\right),0.2\sin\left(0.5t\right),0.15\sin\left(0.7t\right)\right]}^{T},\\ d_{3}={\left[0.1\cos\left(t\right),0.2\cos\left(0.5t\right),0.15\sin\left(0.7t\right)\right]}^{T}. \end{array}$$

The initial quaternions of the follower UAVs are selected as *Q*_1_(0) = [1, 0, 0, 0]^*T*^, *Q*_2_(0) = [0, 1, 0, 0]^*T*^, and *Q*_3_(0) = [0, 0, 1, 0]^*T*^, the initial angular velocities of the follower UAVs are selected as *w*_1_(0) = [0, 0, 1]^*T*^, *w*_2_(0) = [0, 0, 1]^*T*^, and *w*_3_(0) = [0, 0, 1]^*T*^. The initial quaternion of the leader UAV is selected as *Q*_0_(0) = [0, 0, 0, 1]^*T*^, and the angular velocity of the leader UAV is given as*w*_0_(*t*) = [0.1cos(0.2*t*),−0.1sin(0.2*t*),−0.1cos(0.2*t*)]^*T*^.

The article "Event-Triggered Finite-Time Attitude Cooperative Control for Multiple Unmanned Aerial Vehicles" was published in 2022. Journal: Appl Bionics Biomech.

The controller parameters are chosen with *k*_1_ = 1, *k*_2_ = 0.001, *k*_3_ = 0.01, *k*_4_ = 1, *r* = 0.6, *ϕ* = 0.1, *η* = 0.1, and *ρ*_*i*_ = 0.009. The adaptive RBFNN controller parameters are adjusted as *J* = 7, *c*_*i*_ = [−1.5, −1, −0.5, 0, 0.5, 1, 1.5], *σ*_*i*_ = 5, and *A* = diag([0.5 0.5 0.5]^*T*^).

Figures 3 and 4, respectively, show the attitude tracking *Q*_*i*_ and the attitude tracking errors ${\tilde{Q}}_{i}$ of the *i*th UAV,*i* = 1, 2, 3.

Figures 5 and 6, respectively, show the angular velocity tracking *w*_*i*_ and the attitude tracking errors ${\tilde{w}}_{i}$ of the *i*th UAV. From Figures 3–6, it can be seen that the attitude and the angular velocity of all follower UAVs can accurately track the leader UAV over time under the action of the controller (17) and the event-triggered function (23).

Figure 7 shows the evolution process of the measurement error norm of the system, where threshold ‖*e*_*i*_‖_max_ = *k*_3_ + *k*_4_‖*s*_*i*_‖ − *ρ*_*i*_. When the value of ‖*e*_*i*_‖ increases from zero to ‖*e*_*i*_‖_max_, the event is triggered.

Figures 8–10 show the event-triggered time of the UAV *i*, *i* = 1, 2, 3, and the denser part marked by the rectangular box is enlarged. At the event-triggered time of the UAV *i*, the UAV *i* interacts with information and updates the controller.  Figure 11 shows the control torque *u*_*i*_ of the UAV *i*.

From Figures 7–11, it can be seen that the superior performance of the proposed event-triggered control strategy in reducing the energy dissipation of the system and the update frequency of the controller.

The approximation error ‖*ε*_*i*_‖ of the RBFNNs to unknown lumped disturbance *δ*_*i*_ is shown in Figure 12. It can be seen that the RBFNNs can approach *δ*_*i*_ at a faster speed under the action of the adaptive weight update law (23).

## 5. Conclusions

In this paper, a distributed finite time event-triggered control strategy with RBFNNs is proposed for attitude cooperative control of MUAVs. Under the leader-following framework, the tracking errors of attitude converge to zero in finite time, the communication resources is saved and the Zeno behavior is excluded by utilizing the event-triggered scheme. Finally, theory and numerical simulation proof is given for the proposed control law. In the future, we will consider actuator saturation problem by fault-tolerant technology and self-triggered scheme to be used in finite-time control.

The article "Event-Triggered Finite-Time Attitude Cooperative Control for Multiple Unmanned Aerial Vehicles" was published in 2022. Journal: Appl Bionics Biomech.

## Figures and Tables

**Figure 1:** Adaptive RBFNN control.

**Figure 2:** Communication topology.

**Figure 3:** Attitude tracking.

**Figure 4:** Attitude tracking errors.

**Figure 5:** Angular velocity tracking.

**Figure 6:** Angular velocity errors.

**Figure 7:** Variation trend of measurement error norm ‖*e*_*i*_‖ and threshold‖*e*_*i*_‖_max_.

**Figure 8:** Event-triggered time for UAV1.

**Figure 9:** Event-triggered time for UAV2.

**Figure 10:** Event-triggered time for UAV3.

**Figure 11:** Control torques.

**Figure 12:** The RBFNN estimation error ‖*ε*_*i*_‖.

## Data Availability

We have no data to share for this paper.
